The article "Liuwei Dihuang Pill Attenuates Diabetic Nephropathy by Inhibiting Renal Fibrosis via TGF-β/Smad2/3 Pathway" was retracted in 2023. Reasons: unreliable results or conclusions; concerns about the data; concerns about the peer review; concerns about the citations.

# Liuwei Dihuang Pill Attenuates Diabetic Nephropathy by Inhibiting Renal Fibrosis via TGF-*β*/Smad2/3 Pathway

**DOI:** 10.1155/2022/5063636

**Published:** 2022-03-15

**Authors:** Shi Shu, Yue Zhang, Qian Wang, Pengyu Tao, Zhijie Li, Zhongju Xu, Haiying Lu, Lin Shi

**Affiliations:** ^1^Shanghai Punan Hospital of Pudong New District, Shanghai 200125, China; ^2^Basic Medical School, Shanghai University of Traditional Chinese Medicine, Shanghai 200120, China; ^3^Postdoctoral Workstation, Department of Central Laboratory, The Affiliated Taian City Central Hospital of Qingdao University, Taian 271000, China; ^4^Science and Technology Center, Shanghai University of Traditional Chinese Medicine, Shanghai 201203, China; ^5^Shanghai Guanghua Hospital of Integrated Traditional Chinese and Western Medicine, Shanghai 200052, China; ^6^Nursing School, Shanghai University of Traditional Chinese Medicine, Shanghai 200120, China; ^7^Department of Radiology, Affiliated Hospital of Xuzhou Medical University, Xuzhou, 221004 Jiangsu Province, China

## Abstract

Among all the complications of diabetes, diabetic nephropathy is a significant factor causing the end-stage renal disease associated with high death rates. Current treatment fails to produce an ideal outcome. Thus, searching for a new preventive drug is urgently needed. Liuwei Dihuang pill (LDP), a popular ancient Chinese medicine (TCM) prescription, has been applied to treat DN-like syndromes according to TCM theory. Here, we had established an animal model with DN and LDP therapy was put into use to assess its therapeutic effect in vivo. Our data showed that oxidative stress and TGF-*β*/Smad2/3 pathway-induced renal fibrosis could be observed in the DN animal model. However, the treatment of LDP impeded the generation of ROS and attenuated renal fibrosis-related proteins in damaged kidneys through interference in the TGF-*β*/Smad3 pathway. Our results indicated that LDP attenuated oxidative stress, accompanied by preventing the production of renal fibrosis through inhibiting the TGF-*β*/Smad2/3 pathway.

## 1. Introduction

Diabetic nephropathy (DN) is a chronic renal disease characterized by elevated urinary protein and declining glomerular filtration rate caused by diabetes, which also acts as a single factor leading to end-stage renal disease [1]. The WHO releases a report that estimated that 30% of the population worldwide with diabetes will eventually progress into DN that makes the whole society shoulder more economic and health burden [2]. The current treatment toward DN is limited. Although the rational management of food intake and blood glucose control is beneficial to DN, it could not reverse or delay the progress of DN. Thus, exploring the underlying mechanism of DN and developing novel therapy against DN will be beneficial to mankind [3, 4]. Multiple risk factors, such as hypertension, hyperglycemia, obesity, and oxidative stress, are contributing to the occurrence of DN [5]. Among these pathological factors, oxidative stress is considered a vital mediator in the progress of DN [5]. Under hyperglycemia-induced metabolic disturbance, the function of antioxidases is largely inhibited to clear the generation of oxygen radicals. Subsequently, the overwhelming oxidative stress response imposed severe damage on renal tissues [6]. Also, the overwhelming oxidative stress response triggers the activation of various signaling pathways, including the SMAD pathway, MAPK pathway, and protein kinase C (PKC) pathways [7], leading to accumulation and disposition of extracellular matrix ECM [8, 9]. Thus, targeting oxidative stress-mediated renal fibrosis could improve the clinical outcome of DN. There is a wealth of documents on traditional Chinese medicine's (TCM) achievement in healing various diseases. Liuwei Dihuang pill (LDP), a classic herb medicine based on TCM theory, has been widely used to treat patients with diabetes-like symptoms for centuries [10]. Modern scientific research had confirmed the function of LDP manifested in anti-inflammation, reducing blood glucose, and improving renal diseases [11, 12]. In this study, we are going to explore the protective mechanism of LDP on DN with oxidative stress-mediated renal fibrosis. Our results suggest that LDP treatment is effective in attenuating oxidative stress in DN. In addition, LDP treatment also inhibited the renal fibrosis induced by oxidative stress.

## 2. Methods and Materials

### 2.1. Animals

Male C57 BLKS/J db/db mice (5 weeks; body weight 20–22 g) were purchased from the Model Animal Research Information Platform (laboratory animal certificate number: SCXK (Jiang Su) 2010-0001). Mice were kept in single cages and had free access to food and water. The db/db diabetic mice were divided into a normal group (*n* = 16), DN group (*n* = 16), group treated with LDP (*n* = 16), and group treated with valsartan (*n* = 16). The research was authorized by the Animal Ethics Committee of Shanghai University of Traditional Chinese Medicine.

### 2.2. Drug Preparation

The prepared rehmannia root, dogwood, dried yam, alisma, cortex moutan, and white poria are effective ingredients of Liuwei Dihuang pill (LDP) (Beijing Tong Ren Tang Technologies Co, Ltd). Certain amounts of LDPs were melted in distilled water to make aqueous solution (0.675 mg/mL). The same method was also used to make valsartan (Novartis) an aqueous solution (3 mg/mL). The total treatment duration period was 12 weeks. The administration of aqueous solution (1 mL/100 g) is mainly through an intragastric route.

### 2.3. Measurement of Renal Function

Urine samples were collected from mice housed in a metabolic cage for 24 hours and centrifuged to obtain supernatant. Later, these supernatants for each group were used to assay. 24-hour urine protein, blood urea nitrogen, and serum creatinine were assayed; these procedures were all done by HITACHI automatic biochemical instrument. The supernatant used to determine the concentration of SOD and MDA was collected according to the following steps: the 15 mg kidney tissues of each group were harvested and cleaned with cold saline, later homogenized by vibrating homogenizer with cold saline. Finally, the concentration of SOD and MDA in the supernatant was detected by a following protocol provided by the SOD kit and MDA kit, respectively (Nanjing Jiancheng Biological Technology).

### 2.4. HE Staining

Animals were anesthetized by pentobarbital sodium (3%, 0.2 mL/100 g). The kidneys were then removed and measured. Hematoxylin-eosin staining (HE) is performed as follows: the renal cortex was harvested and fixed in 10% neutral buffered formalin solution, dehydrated, embedded, and finally made into a sample of 3 *μ*m thick before being observed under light microscopy. Kidney tissues were also made into cubes (1 mm × 1 mm × 1 mm) for electron microscope use after being fixed in 2% glutaraldehyde, washed with 0.1 M phosphate buffer, fixed in 1% osmic acid, and rinsed with phosphate buffer (Model TECNAI-12, Netherlands).

### 2.5. Western Blot Analysis

According to the protocol, an appropriate amount of renal tissue was harvested and incubated in a tube containing PMSF, RIPA, and phosphatase inhibitors, later homogenated with ultrasound (15,000 r/min for 20 min at 4°C), and finally centrifuged to obtain the supernatant storing at -80°C. The quantification of protein solution was determined by BCA kit. The Western blot analysis is carried out through electrophoresis, membrane transfer, sealing, TBST washing, first antibody incubation, TBST washing, secondary antibody incubation, TBST washing, adding developer, and exposure strip. The antibodies (Cell Signaling Company) are used as follows: p38 (9212), p-p38 (4511), TGF-*Β* (3712), Erk (4695), p-Erk (4370), Smad2 (5339), p-Smad2 (3108), Smad3 (9513), p-Smad3 (9520), and GAPDH (2118s).

### 2.6. Statistical Analysis

The data were presented as mean ± standard deviation (SD). SPSS 23.0 was employed to analyze all data. One-way analysis of variance (ANOVA) test was used to compare multiple sample groups, and *p* < 0.05 was considered statistically significant.

## 3. Results

### 3.1. LDP Improved Biochemical Indicators

Compared with the NC group, the levels of 24TP, BUN, and Cr went through a sharp increase in the DN group (*p* < 0.05, Figures 1(b), 1(d), and 1(e)). However, their levels reduced after being treated with LDP. The DN group was characterized by polydipsia, polyphagia, polyuria, fur loss, weight loss, cold limbs, and lag of responses. But we observed that the symptoms mentioned above were improved in the LDP group.

### 3.2. LDP Prevents Oxidative Stress

The excessive production of oxygen-free radicals served as a vital factor in the progression of DN. SOD, MDA, and NOS are sensitive indicators of oxidative stress. Compared with the NC group, the levels of NOS and SOD were significantly decreased while MDA was upregulated in the DN group. But the levels of SOD and NOS were elevated as well as the reduction in the expression of MDA after administration of LDP (Figures 1(c) and 1(f)). Therefore, the results have confirmed that LDP exerts renal protection against oxidative stress mainly through increasing the production of SOD and NOS as well as inhibiting the generation of MDA.

### 3.3. LDP Attenuated Renal Pathology

The glomerular hypertrophy, basement membrane thickening, and mesangial matrix expansion are considered as the typical changes in DN pathology. We performed an experiment on the efficacy of LDP against DN. Kidney coefficient is used to measure the volume of the kidney. Compared with the NC group, kidney coefficients are increased in the DN group but rescued after being treated with LDP (Figure 2(e)), which indicates that kidney hypertrophy can be relieved by LDP therapy. We also conduct HE staining of kidney tissues to examine the renal glomerular structure. HE staining revealed that the glomerular volume in the DN group was larger than that in the NC group, accompanied by the increasing number of cells and proliferation of mesangial matrix (Figure 2(a)). By contrast, less change was observed in the glomerular structure from the LDP group (Figure 2(c)). In addition, we also examined the renal tissues from the DN group by employing electron microscopy. Podocyte swelling, foot process flattening, and fusion were observed in the DN group, which were significantly attenuated in LDP groups (Figures 2(c) and 2(d)). Therefore, the results have confirmed that LDP therapy exerts renal protection against DN mainly through maintaining the intact glomerular structure and protecting podocyte from high glucose.

### 3.4. LDL Inhibited Oxidative Stress-Induced Renal Fibrosis via Regulating the TGF-*β*/Smad2/3 Pathway

The TGF-*β*/Smad2/3 pathway acts as a significant factor contributing to renal fibrosis; thus, targeting the TGF-*β*/Smad2/3 pathway could suppress profibrotic response in DN. Western blot results revealed that compared with normal mice, there was upregulation of TGF-*β* RI and RII in DN mice (Figure 3(a)), but it was reduced by LDP therapy. In addition, we observed that the expressions of Smad2 and Smad3 protein were no different among all groups, but the phosphorylation of Smad2 and Smad3 protein was enhanced in DN (Figures 3(b) and 3(c)), proving that the TGF-*β*/Smad2/3 pathway was activated in DN, which was inhibited by the LDP therapy. Thus, we have proven that LDP played a suppressive role in renal fibrosis through prohibiting the TGF-*β*/Smad2/3 pathway.

### 3.5. LDL Inhibited Oxidative Stress-Induced Inflammation via Regulating the MAPK Pathway

The role of inflammation induced by oxidative stress in DN has gained attention from scientific community. The activation of inflammatory response also stimulated the upregulation of the TGF-*β*/Smad2/3 pathway leading to renal fibrosis in DN. The MAPK pathway is considered a key mediator in inflammation. Western blot results suggested that the expressions of Erk and p38 protein were no different among all groups, but the phosphorylation of Erk and p38 protein was upregulated in the DN group (Figures 4(b) and 4(d)), compared with the NC group, confirming that the activation of inflammation contributed to DN. But it was suppressed by the therapy of LDP. A similar effect was gained in the valsartan group. Thus, we have proven that LDP owns the ability to protect the kidney against inflammation in DN.

## 4. Discussion

Diabetic nephropathy (DN) is a metabolic disease that refers to typical pathological changes characterized by proliferation in the number of mesangial cells, basement membrane thickening, and extracellular matrix expansion [13]. Although current treatment including strictly controlling blood glucose levels, limiting protein intake, and altering lifestyle can control DN, these methods do not offer enough protection against DN [14]. Traditional Chinese medicine has made significant progress in DN remedy. High blood glucose is one of the typical clinical features in DN. As the disease progresses, high blood glucose leads to the apoptosis of podocyte, which is the main cause of massive proteinuria. When it comes to end-stage renal disease, the kidney function is in poor condition as well as a serious renal pathology. However, the bioindicators and renal pathology were alleviated by LDP therapy. The results indicated that LDP therapy could reduce the blood glucose levels, improve renal function, and offer renal protection against DN.

The oxidative stress response is an important mechanism contributing to DN [15]. SOD and NOS are two of the most active antioxidant enzymes that serve a key role in removing ROS, while MDA is positively correlated with oxidative stress damage [16]. The high-glucose-induced generation of ROS impairs the antioxidant enzyme system via downregulation of SOD and upregulation of MDA. The impaired antioxidant enzyme system causes more generation of ROS leading to continuous oxidative stress that damages kidney tissues [17]. Thus, it is noted that a vicious oxidative stress caused by ROS imposes damage on the kidney in DN, and the reduction of ROS generation is undoubtedly an effective treatment for DN [17]. In the present study, we performed the experiment of LDP mediated-antioxidative stress regulatory mechanism in diabetic mice. The results revealed that LDP therapy evidently raised the level of SOD and NOS and decreased the level of MDA. It implied that LDP therapy can attenuate oxidative stress by restoring the activity of SOD and NOS and inhibiting the activation of MDA.

Oxidative stress and renal fibrosis are two important mechanisms contributing to DN [17]. Moreover, the enhanced expression of the TGF-*β*/Smad2/3 and MAPK pathway activated by oxidative stress was shown to occur in diabetic mice. TGF-*β* served as a vital regulator in renal fibrosis. Under the influence of diabetic condition, a large amount of ROS generated inside mesangial cells stimulates the generation of ECM and inhibits its degradation via enhancing the expression of TGF-*β* to cause renal fibrosis [18, 19], because (1) ROS stimulates the activation of TGF-*β*/Smad pathway to accelerate the formation of renal fibrosis and (2) TGF-*β* activates Ang II to be responsible for renal fibrosis. The MAPK pathway is a key downstream effector of ROS, which has a strong link to renal fibrosis [20]. The phosphorylation of p38 and Erk protein induced by ROS is involved in the generation and accumulation of ECM in DN [21]. The activation of p38 and Erk protein promotes TGF-*β* to bind to TGF-*β*. Type I and type II receptors bind on the cell membrane [22]. Subsequently, phosphorylated Smad2/3 in the cytoplasm leads to the activation of the TGF-*β*/Smad signaling pathway [23]. Our data confirmed that the stimulation of the TGF-*β*/Smad2/3 and MAPK pathway acting as a vital regulator in the expression and secretion of ECM eventually leads to renal fibrosis in DN.

To further study the therapeutic efficacy of LDP therapy against renal fibrosis, we had constructed an animal DN model with renal fibrosis by using db/db mice. Interestingly, as our results revealed that LDP therapy evidently suppressed the expression of TGF-*β* as well as the high phosphorylation of SMAD2/3 in renal tissues. The high phosphorylation of p38 and Erk was also observed in kidney tissues but could be reduced by LDP treatment, which inhibited the MAPK signaling pathways in an effective way. To sum up, these data suggested that LDP treatment can attenuate renal fibrosis in the DN model mainly through inhibiting the TGF-*β*/Smad2/3 pathway and MAPK pathway.

In conclusion, our study has demonstrated the protective mechanism of LDP therapy on the DN model. LDP therapy can significantly reduce the blood glucose level and ameliorate renal damages. LDP also can suppress the oxidative stress response and formation of renal fibrosis by inhibiting the TGF-*β*/Smad2/3 pathway and MAPK pathway.

## Figures and Tables

**Figure 1:** The effect of LDP therapy on renal function in DN via decreasing the level of urine protein (b), Cr (d), and BUN (e) as well as inhibiting oxidative stress via decreasing the level of MDA (c) and enhancing the level of SOD (f).

**Figure 2:** The effect of LDP therapy on renal pathology in DN. The enlarged glomerular volume and increased number of mesangial cells in the DN group (a). The podocyte swelling, foot process flattening, and fusion were relieved by LDP and valsartan (b, d).

**Figure 3:** The LDP therapy reduced renal fibrosis in DN by blocking the expression of TGF-*β* RI, TGF-*β* RII (a), phosphorylated Smad2 (b), and phosphorylated Smad3 (c).

**Figure 4:** The effect of LDP therapy blocks the MAPK pathway in DN by reducing the expression of phosphorylated Erk (b) and p38 (d).

## Data Availability

The data presented in the study may be made available from the corresponding author upon reasonable request.
